# Regulatory Mechanism of circEIF4G2 Targeting miR-26a in Acute Myocardial Infarction

**DOI:** 10.1155/2022/5308372

**Published:** 2022-03-16

**Authors:** Zaiyong Zhang, Jianhao Li, Cheng Long, Yuanyuan Han, Jun Fan, Afzal Misrani, Xiangyu Ji

**Affiliations:** ^1^Department of Cardiology, Panyu Central Hospital, Guangzhou 511400, China; ^2^Cardiovascular Institute of Panyu District, Guangzhou 511400, China; ^3^South China Normal University-Panyu Central Hospital Joint Laboratory of Translational Medical Research, Panyu Central Hospital, Guangzhou 511400, China; ^4^School of Life Sciences, South China Normal University, Guangzhou 510630, China; ^5^Department of Radiology, Panyu Central Hospital, Guangzhou 511400, China

## Abstract

**Background:**

Acute myocardial infarction (AMI) involves a series of complex cellular and molecular events, including circular RNAs (circRNAs), microRNAs (miRNAs) and other noncoding RNAs.

**Objective:**

In this study, the regulation mechanism of circEIF4G2 acting on miR-26a on HUVECs (Human Umbilical Vein Endothelial Cells) proliferation, cell cycle and angiogenesis ability was mainly explored in the vascular endothelial growth factor induced (VEGF-induced) angiogenesis model.

**Methods:**

VEGF induced HUVECs angiogenesis model was constructed, and the expression of circEIF4G2 and miR-26a in VEGF model was detected by qRT-PCR. When circEIF4G2 and miR-26a were knocked down or overexpressed in HUVECs, qRT-PCR was used to detect the expression of circEIF4G2 and miR-26a, CCK-8 was used to detect cell proliferation, flow cytometry was used to detect the cell cycle transition of HUVECs, and cell formation experiment was used to detect the ability of angiogenesis. MiRanda database and Targetscan predicted the binding site of circEIF4G2 and miR-26a, lucifase reporting assay and RNA pull down assay verified the interaction between circEIF4G2 and miR-26a.

**Results:**

After HUVECs were treated with VEGF, circEIF4G2 was significantly upregulated. After circEIF4G2 was knocked down, the proliferation and angiogenesis of HUVECs cells were decreased, and the process of cell cycle G0/G1 phase was blocked. The overexpression of miR-26a reduced the proliferation and angiogenesis of HUVECs cells and blocked the cell cycle progression of G0/G1 phase. Double lucifase reporter gene assay verified that circEIF4G2 could directly interact with miR-26a through the binding site, and RNA Pull down assay further verified the interaction between circEIF4G2 and miR-26a. When circEIF4G2 and miR-26a were knocked down simultaneously in HUVECs, it was found that knocking down miR-26a could reverse the inhibition of circEIF4G2 on cell proliferation, cycle and angiogenesis.

**Conclusion:**

In the VEGF model, circEIF4G2 was highly expressed and miR-26a was low expressed. MiR-26a regulates HUVECs proliferation, cycle and angiogenesis by targeting circEIF4G2.

## 1. Introduction

Acute myocardial infarction (AMI) is a common cardiovascular disease. How to maximize the benefits of patients is the direction that needs to be explored and studied in the field of AMI diagnosis and treatment [1–3]. AMI involves a series of complex cellular and molecular events, and various molecules in cells coordinate with each other to respond to AMI. Studies have shown that noncoding RNAs (ncRNAs) such as circRNA, miRNA and long noncoding RNA (lncRNA) can play a key role in the occurrence and progression of heart disease [4, 5]. Noncoding RNAs usually regulate protein gene expression through competing endogenous RNAs (ceRNAs) and affect disease progression [6].

CircRNA is a novel type of RNA whose unique structure is generated by a 3′–5′ end joining event (reverse splicing). Once circular RNA is produced, it may remain in the nucleus as observed with intron-retaining multiexon rings, and most of it will be exported to the cytoplasm. Regardless of location, the unique structure of circRNAs ensures that the molecule is protected from exonuclear dissolution decay and thus remains very stable [7]. Apoptosis of AMI cells involves a variety of apoptosis signals, including cytokines, hypoxia, increased oxidative stress and DNA damage, and circrNa-miRNA-mRNA axis is no exception [8]. Li et al. [9] suggested that circNCX1 gene transcribed from sodium/calcium exchanger 1 (ncx1) plays a key role in the regulation of cardiomyocyte apoptosis by regulating miR-133a-3p and its target cell death inducing protein CDIP1. Liu et al. [10] suggested that after circZNF609 was knocked out, endothelial cell migration level was increased and resistance to oxidative stress was enhanced, while overexpressed circZNF609 showed the opposite effect. CircZNF609 inhibited the activity of miR-133a-3p and increased the expression level of MEF2A, which could inhibit the effect of circZNF609 silencing on endothelial cells. Myocardial cell proliferation and neovascularization are two major biological processes of AMI cardiac repair. The synergistic effect between the two is essential for cardiac regeneration and repair, and circRNA is also involved [11].

MiRNA is a large class of small noncoding RNA molecules that can be widely recognized early [12, 13]. The vast majority of these molecules originate from noncoding genes with a length of about 22nt, and were thought to be functionally antisense modulators of other RNAs in the early stage [14]. MiRNA genes are often expressed singly, but many occur in clusters of 2–7 genes with small intervention sequences. Experimental results suggest that these genes exhibit simultaneous transcription, suggesting that they may be controlled by common upstream gene sequences [15, 16]. Other miRNA genes were excised from introns of protein-coding genes [17, 18] and exons of noncoding genes [19], or even from 3′-UTR of protein-coding genes [20]. In mammalian genomes, miRNAs may also be found in repetitive regions. However, translocation factors may be involved in the generation of new miRNAS [21]. MiRNA can inhibit the mRNA translation of target genes on the basis of certain base pairing, thus participating in the regulation of target protein expression. In recent years, a number of studies have shown that some miRNAs protect the heart by going up or down by altering key signaling elements. These effects play a protective role through miRNAs and/or antagonists in ischemic preconditioning, regulation of heat shock proteins, antihypoxia and pharmacological preconditioning [22].

In this study, the molecular regulatory mechanism of AMI related circRNA was studied, providing a new theoretical basis for the molecular mechanism of myocardial infarction, and thus providing a new intervention strategy for the treatment of myocardial infarction.

## 2. Materials and Methods

### 2.1. Abbreviation and Full Title

All abbreviations and full titles are shown in Table 1.

### 2.2. Establishment of VEGF-Induced HUVECs Angiogenesis Model

HUVECs were cultured with DMEM medium containing 10% FBS. HUVECs were treated with VEGF to promote angiogenesis, and VEGF induced angiogenesis model of HUVECs were established.

### 2.3. Transfection

SiRNA for circEIF4G2, mimics and siRNA for miR-26a and NC were purchased from Shanghai Jikai gene Chemical Technology Co., Ltd. Transfection was performed according to the instructions of Lipofectamine 2000 Reagent (Shanghai Qifa Experimental Reagent Co., Ltd.). The detailed operations were as follows. 24 well cell culture plate was prepared and cells were cultured in DMEM medium with 10% FBS. The corresponding inoculation density was controlled as 2 × 10^4^ per well for one day. It was observed that when the cells were fully fused, the culture medium was removed and fully rinsed with the phosphate buffer. Then, 0.3 mL OPTI-MEM was added into each well, and the culture was transferred to standard conditions for full cultivation. 1 *μ*L lipofectamine 2000 reagent was diluted by the above medium and diluted 50 times to get 50 *μ*L. The reagent was placed at room temperature for 10 minutes. 1 *μ*L of 20 *μ*M miRNA mimics, inhibitors, and 0.5 *μ*g plasmid were added to OPTI-MEM medium, and put it at room temperature for 5 minutes. Concentrations of miRNA mimics and inhibitors were eventually adjusted to 50 nM. They were mixed with lipofectamine 2000 reagent which diluted 50 times and put at room temperature for 20 minutes. 0.1 mL of transfection mixture was added into each well. After proper mixing, it was cultured under standard environmental conditions for 5 hours. Finally, the transfection reagent was moved away and DMEM medium with fresh 10% FBS was added.

### 2.4. qRT-PCR

Total RNA was extracted from HUVECs, and the RNA was reversely transcribed into cDNA using reverse transcriptase (Thermo, USA), which was used as a template for PCR amplification. According to the design principle of real-time quantitative PCR primers, circRNA sequences were downloaded from circBase database and PCR primers designed for hSA_CIRC_0021245 (circEIF4G2) reverse splices were as follows:

  circEIF4G2:
  F:CAAGTCATGTTCATGCCCTGA, R:TCCATGTCATAGAAGTGCACA
  EIF4G2:
  F:CCACAAGTGACAACTTCATGC, R:TCTGAAATGCTCACCAGCTCT
 
*β*-Actin:
  F:CATGTACGTTGCTATCCAGGC, R:CTCCTTAATGTCACGCACGAT

### 2.5. CCK-8

HUVECs, which were transfected for 48 hours were inoculated in a 96-well culture plate with 1.5 × 103 cells/mL, 100 *µ*L per well. The 96-well plates were placed in an incubator for 1, 2, 3, 4, and 5 days, respectively (the blank control group was medium without cells). 10 *µ*L CCK-8 reagent (APExBIO, USA) was added to each well and cultured in an incubator for 4 hours. At the absorption wavelength of 450 nm, the absorbance value of each well was recorded with a microplate reader, and the growth curve of cells was plotted.

### 2.6. Flow Cytometry

Transfected HUVECs for 48 hours after digested with trypsin, terminated digestion and centrifuged. The cells were washed with phosphate buffer twice, centrifuged at 1000 rpm for 5 minutes, and collected. Suspended cells by adding 500 *µ*L binding buffer (Shanghai QianChen Biotechnology Co., Ltd.). Annexinv-fitc (Shanghai Qianchen Biotechnology Co., Ltd.) was added to 500 *µ*L cell suspension, mixed and incubated for 15 minutes. 5 *µ*L Propidium Iodide dye (Shanghai Qianchen Biological Co., Ltd.) was added to cell suspension, mixed well, and incubated for 15 minutes under dark conditions. The fluorescence intensity was determined by flow cytometry.

### 2.7. Tube Formation Assay

Matrigel glue was put on ice to melt, and the gun head and 96-well plate were put at −20°C refrigerator to precool. The precooled gun heads were used to take Matrigel glue 100 *µ*L/well and added it to the precooled 96 well plate. Pay attention to avoid the formation of bubbles. Place it on ice for 5 minutes to make the Matrigel level, and then put the plate into 37°C cell incubator for 30 minutes to solidify the gel. The 100 *µ*L HUVECs (1.5 × 104 cells/well) were added to the well containing Matrigel gel. At the same time, the tested compounds diluted into different concentrations with M199 medium and DMSO control were added and cultured at 37°C for 8 hours. Observed and photographed under a microscope. Five fields were randomly selected to take photos and image Pro Plus software was used to calculate the length of cavity formation.

### 2.8. Double Luciferase Reporting Experiment

The luciferase reaction reagent (5 mL + 1 vial) were dissolved, repacked and stored it under dark conditions. Mix as required to obtain luciferase reaction reagent II, and then stored it in dark after subpackaging. Lysis buffer and double distilled water were mixed for treatment. After transfecting for 48 hours, the culture medium was absorbed and discarded, and the cells were fully rinsed with phosphate buffer. Then, the cells were placed in the wells of cell lysis buffer at room temperature for 10 minutes. After full pyrolysis, took the pyrolysis solution and added it into the sterilized centrifuge tube. Then centrifuged at high speed at 4°C for 10 minutes, and took the supernatant for determination. Turn on the fluorometer according to relevant operating specifications, with an interval of 2 seconds and test for 10 seconds. Taking out the preserved reaction reagent and balanced it at room temperature. Then took out 20 *µ*L of sample, added 100 *µ*L of luciferase reaction reagent (Hanheng Bioengineering (Shanghai) Co., Ltd.), and detected RLU after appropriate mixing. The control test group was reporter gene cell lysate. Taking an appropriate amount of luciferase reaction reagent II and balanced it to room temperature. After the above tests were completed, then added 0.1 mL of luciferase II into each tube, and detected RLU after sufficient mixing. Set luciferase as the internal parameter, divided its RLU value by the RLU value determined by detection, and reflected the activation degree of the target gene based on the obtained results.

### 2.9. RNA Pull down

Biotin labeled wt-miR-26a and mut-miR-26a RNA fragments were synthesized and transfected into HUVECs using Lipofectamine 2000 (Thermo Fisher Scientific (Shanghai) Co., Ltd.), respectively. After 48 hours of transfection, the 100 *µ*L RIP solution which containing protease inhibitor (Roche) and RNase inhibitor (Promega) were added for cracking according to Magna RIP Kit (Millipore). Cell lysates were collected and incubated with RNase-free BSA and TRNA-coated streptavidin agarose beads, and ice bath for 2 hours. It was centrifuged and washed with buffer. Then according to the kit instructions, RNA was extracted using TRIzol Regent (Invitrogen), and circEIF4G2 was detected by qRT-PCR. The antagonist miR-26a probe was set as a negative control.

### 2.10. Statistical Analysis

Statistical analysis was performed by using the GraphPad Prism 8.0 software. The *t*-test was used between the two groups, ANOVA between multiple groups, and *P* < 0.05 was statistically significant. Repeat three times for each set.

## 3. Results

### 3.1. Expression of circEIF4G2 in the Angiogenesis Model of HUVECs

We have known the expression of circEIF4G2 and miR-26a in peripheral blood of patients with myocardial infarction through previous studies, but their regulatory mechanism in myocardial infarction is still unclear. In order to investigate the role of circEIF4G2 in promoting angiogenesis, HUVECs were treated with corresponding VEGF, and the expression of circEIF4G2 was detected by amplification method. It was found that circEIF4G2 was upregulated by 7.54 ± 0.53 in VEGF treatment group, which was significantly different from that in control group (Figure 1(a)). Compared with the control group, the expression of miR-26a in VEGF treatment group was down regulated (Figure 1(b)). These results suggest that circEIF4G2 may be regulated by angiogenic factor VEGF.

### 3.2. Effects of Knockdown of circEIF4G2 on Proliferation, Cell Cycle, and Angiogenesis of HUVECs

After knockdown circEIF4G2 with siRNA, the proliferation ability of HUVECs was detected by CCK-8. The proliferation ability of the interference group decreased significantly from day 3 (Figure 2(a)). Flow cytometry was used to detect the cell cycle process of HUVECs after circEIF4G2 knockdown. The results showed that the G1/G0 phase was blocked after knockdown of circEIF4G2 (48% and 66%, respectively) (Figure 2(b)). The results of angiogenesis experiment showed that knockdown of circEIF4G2 significantly inhibited the angiogenesis of HUVECs, and the complete vascular network structure could not be obtained (Figure 2(c)). These results suggest that knockdown of circEIF4G2 inhibits the proliferation, cycle progression and angiogenesis of HUVECs.

### 3.3. Effects of Overexpression or Knockdown of miR-26a on Proliferation, Cycle, and Angiogenesis of HUVECs

After miR-26a was overexpressed or knocked down, the expression rates of miR-26a and circEIF4G2 were detected by qRT-PCR. When miR-26a was overexpressed in HUVECs, compared with the control group, the expression of miR-26a was upregulated (Figure 3(a)), while the expression of circEIF4G2 was downregulated (Figure 3(b)). When miR-26a was knocked down in HUVECs, compared with the control group, the expression of miR-26a was downregulated (Figure 3(c)), while the expression of circEIF4G2 was upregulated (Figure 3(d)). After miR-26a was overexpressed by transfecting miR-26a mimics into HUVECs, the proliferation ability, cell cycle progression and angiogenesis ability of HUVECs were detected. Compared with the control group, its proliferation ability was reduced (Figure 3(e)). The cell cycle was also arrested in G1/G0 phase (47% and 80%, respectively) (Figure 3(f)). The results of angiogenesis experiment showed that overexpression of miR-26a significantly inhibited the angiogenesis ability of HUVECs, and the complete vascular network structure could not be obtained (Figure 3(g)). This suggests that overexpression of miR-26a also inhibits HUVECs proliferation, cycle progression and angiogenesis.

### 3.4. circEIF4G2 Interacts with miR-26a

MiRanda database and Targetscan were used to predict the binding sites of circEIF4G2 and miR-26a, and the results showed that circEIF4G2 had binding sites with miR-26a (Figure 4(a)). The direct interaction between circEIF4G2 and miR-26a was verified by dual lucifase reporter gene and RNA-pull down (RIP) assay. The results showed that when wild-type circEIF4G2 was cotransfected with miR-26a mimics, the fluorescence value of lucifase reporter gene was decreased. After the combination of circEIF4G2 mutant with miR-26a, the fluorescence value increased, and there was no difference between the two groups (Figure 4(b)). The results indicated that circEIF4G2 could directly interact with miR-26a through binding sites. To further verify the interaction between circEIF4G2 and miR-26a, HUVECs cells were transfected with biotin marking the wild type 3′ end and mutant 3′ end of miR-26a mimics. RNA molecules bound to biotin-labeled miR-26a were captured by magnetic beads coated with streptomycin, and the abundance of circEIF4G2 was detected by qPCR. The results showed that circEIF4G2 molecules were significantly enriched in IP group compared with the control group (Figure 4(c)). These results indicated that circEIF4G2 had direct interaction with miR-26a.

### 3.5. miR-26a Is an Important Component that Mediates circEIF4G2 to Promote HUVECs Proliferation, Cell Cycle, and Angiogenesis

The plasmid with knockdown miR-26a and knockdown circEIF4G2 were cotransfected into HUVECs. The experimental groups were NC plasmid group, si circEIF4G2 plasmid group and si miR-26a + si circEIF4G2 plasmid group. The proliferation ability of the si circEIF4G2 plasmid group and the si miR-26a + si circEIF4G2 plasmid group were significantly reduced compared with the control group. Moreover, the cell proliferation ability of the si circEIF4G2 plasmid group was weaker than that of the si miR-26a + si circEIF4G2 plasmid group (Figure 5(a)). Compared with the control group, the cell cycle of the si circEIF4G2 plasmid group and the si miR-26a + si circEIF4G2 plasmid group were arrested in G1/G0 phase. Moreover, more cells were blocked in G1/G0 phase in the si circEIF4G2 plasmid group than in the si miR-26a + si circEIF4G2 plasmid group (Figure 5(b)). In the angiogenesis experiment, compared with the control group, the si circEIF4G2 plasmid group and the si miR-26a + si circEIF4G2 plasmid group could not obtain the complete vascular network structure. However, the ability of promoting angiogenesis in the si miR-26a + si circEIF4G2 plasmid group was stronger than that in the si circEIF4G2 plasmid group (Figure 5(c)). The above results suggest that miR-26a knockdown can partially reverse the inhibitory effects of circEIF4G2 knockdown on the proliferation, cell cycle and angiopoiesis of HUVECs. It is suggested that miR-26a is an important component that mediates circEIF4G2 to promote HUVECs proliferation, cell cycle and angiogenesis.

## 4. Discussion

Acute myocardial infarction is a common heart disease. In the process of treatment, the myocardial blood supply in the ischemic area should be restored as soon as possible, which is of great significance to improve the prognosis [23, 24]. The proliferation and neovascularization of myocardial cell are two major biological processes of AMI cardiac repair. The synergistic effect between the two is essential for cardiac regeneration and repair, and circRNA is also involved [11]. Regulating circRNA expression may be a potential strategy to promote cardiac function and remodeling after myocardial infarction.

Angiogenesis is a complex process of producing new capillaries. The regulation of angiogenesis includes endothelial cells' proliferation, migration, basement membrane rupture and relates growth factors, such as VEGF and FGF-2 [25–27]. Inhibiting the proliferation of this type of cells can improve the antiangiogenic activity. AMI caused severe damage to the coronary microcirculation, resulting in the collapse of blood vessels and thinning of capillaries in the infarct area. Tissue repair after MI involves a powerful angiogenic response that begins at the infarct boundary and extends to the necrotic infarct core. Advances in several areas have provided novel mechanologic understanding of postinfarction angiogenesis and how it may be targeted to improve cardiac function after MI. Currently, it is generally accepted that angiogenesis is derived from tissue-derived signaling pathways, among which VEGF pathway is the most important [28, 29]. This factor is a glycoprotein that play an important role in promoting angiogenesis by promoting endothelial cell growth. VEGF-b, VEGF-c, and VEGF-d are the main members of the VEGF family. VEGF-c and VEGF-d are mainly involved in the regulation of lymphangiogenesis. VEGF downstream signaling pathways include JAK2, PLC*γ*1, etc., which can regulate the proliferation of vascular endothelial cells based on these pathways. In addition, Src and FAK signaling pathways can promote their migration, while JAK2 and Akt pathways are closely related to their apoptosis. According to Garikipati's analysis [30], overexpression of circFndc3b in cardiac endothelial cells could increase the expression of VEGF-A, enhance the angiogenesis activity, and reduced apoptosis of cardiomyocytes and endothelial cells. After myocardial infarction, adeno-associated virus-9 mediated myocardial overexpression of circFndc3b reduced myocardial apoptosis, enhances neovascularization and improved left ventricular function. CircFndc3b interacts with fused RNA-binding proteins in sarcomas to regulate VEGF expression and signal transduction. Therefore, understanding the mechanisms underlying the improvement of infarct angiogenesis may yield multiple therapeutic opportunities. During preclinical development, possible angiogenesis promotion strategies will be tested to provide mechanistic insights into treatment options for myocardial infarction patients.

In our study, HUVECs were treated with VEGF to establish the angiogenesis promoting model, and the effect of circRNA on angiogenesis of vascular endothelial cells was discussed. qPCR showed that the expression level of circEIF4G2 was significantly upregulated after VEGF induction. After siRNA knockdown circEIF4G2, CCK-8 detected the proliferation of HUVECs. It was found that down regulating circEIF4G2 could block the proliferation of HUVECs stimulated by VEGF. The detection of cell cycle suggests that interference with circEIF4G2 may lead to the weakening of cell proliferation and angiogenesis by blocking the process of G0/G1 phase in the metaphase of HUVECs. In the cell model, miR-26a mimics were transfected into HUVECs, and overexpression of miR-26a obtained a similar functional phenotype. This negative correlation between circEIF4G2 and miR-26a in expression level and functional phenotype. Next, the results of double luciferase reporter gene experiment and RNA pull down experiment showed that there was a direct interaction between circEIF4G2 and miR-26a. SiRNA targeting miR-26a was co-infected with circEIF4G2 interfering cells. It was found that knockdown of miR-26a could partially reverse the inhibitory effects of knockdown of circEIF4G2 on the proliferation, cycle and angiogenesis of HUVECs.

This article has its limitations. Firstly, we constructed a VEGF-induced angiogenesis model, and verified the regulatory effect of circEIF4G2 and miR-26a on the VEGF-induced model and the interaction between circEIF4G2 and miR-26a. However, the signal pathway of its action has not been studied. We will continue to improve it in future studies.

## 5. Conclusion

After HUVECs were treated with the VEGF, the expression of circEIF4G2 was significantly upregulated and the expression of miR-26a was downregulated. miR-26a is an important component that mediates circEIF4G2 to promote HUVECs proliferation, cell cycle and angiogenesis. These results provide a new theoretical basis for the molecular mechanism of myocardial infarction and provide a new intervention strategy for the treatment of myocardial infarction.

## Figures and Tables

**Figure 1:** CircEIF4G2 was upregulated and miR-26a was downregulated. (a) The expression levels of circEIF4G2. (b) The expression levels of miR-26a.  ^*∗*^ ^*∗*^ ^*∗*^*P* < 0.001 vs. control group.

**Figure 2:** Downregulation of circEIF4G2 inhibited HUVECs proliferation, blocked cell cycle and inhibited angiogenesis. (a) The expression levels of circEIF4G2 were detected by qRT-PCR after knockdown of circEIF4G2. (b) CCK-8 was used to detect cell proliferation after knockdown of circEIF4G2. (c) Cell cycle transformation was detected by flow cytometry after knockdown of circEIF4G2. (d) Detection of angiogenesis by cell formation assay after knockdown of circEIF4G2.  ^*∗*^ ^*∗*^*P* < 0.01 and  ^*∗*^ ^*∗*^ ^*∗*^*P* < 0.001 vs. control group.

**Figure 3:** Overexpression of miR-26a inhibited HUVECs proliferation, blocked cell cycle, and inhibited angiogenesis. (a, b) The expression levels of miR-26a and circEIF4G2 were detected by qRT-PCR after overexpressing miR-26a. (c, d) The expression levels of miR-26a and circEIF4G2 were detected by qRT-PCR after knockdown of miR-26a. (e) The proliferation ability of HUVECs were detected by CCK-8 after overexpression of miR-26a. (f) The cell cycle progression of HUVECs was detected by flow cytometry after overexpression of miR-26a. (g) Angiogenesis of HUVECs was detected by cell formation assay after overexpression of miR-26a.  ^*∗*^ ^*∗*^*P* < 0.01 and  ^*∗*^ ^*∗*^ ^*∗*^*P* < 0.001 vs. NC group.

**Figure 4:** CircEIF4G2 can bind to miR-26a directly. (a) MiRanda database and Targetscan predicted the binding sites of circEIF4G2 and miR-26a. (b) Lucifase reporter gene assay verified that circEIF4G2 could directly target miR-26a. (c) Detection of interaction between circEIF4G2 and miR-26a by RNA pulldown assay.  ^*∗*^ ^*∗*^*P* < 0.01 and  ^*∗*^ ^*∗*^ ^*∗*^*P* < 0.001 vs. NC group.

**Figure 5:** Downregulation of miR-26a partially reversed the inhibition of circEIF4G2 downregulation on proliferation, cell cycle and angiogenesis of HUVECs. (a) The proliferation ability of cells was detected by CCK-8. (b) The cycle progression of HUVECs were detected by flow cytometry. (c) The angiogenesis was detected by cell formation assay.  ^*∗*^*P* < 0.05 and  ^*∗*^ ^*∗*^*P* < 0.01 vs. control group. ^#^*P* < 0.05 vs. si circEIF4G2 group.

**Table 1:** Abbreviation and full title.

Abbreviation	Full title
AMI	Acute myocardial infarction
circRNAs	Circular RNAs
miRNAs	MicroRNAs
HUVECs	Human umbilical vein endothelial cells
VEGF	Vascular endothelial growth factor
ncRNAs	Noncoding RNAs
lncRNA	Long noncoding RNA
ceRNAs	Competing endogenous RNAs
FBS	Foetal bovine serum

## Data Availability

The data used to support the findings of this study are included within the article.
